# Targeted temperature management in traumatic brain injury

**DOI:** 10.1186/s40560-016-0137-4

**Published:** 2016-04-27

**Authors:** Shoji Yokobori, Hiroyuki Yokota

**Affiliations:** Department of Emergency and Critical Care Medicine, Nippon Medical School, 1-1-5, Sendagi, Bunkyo-Ku, Tokyo 113-8603 Japan

**Keywords:** Targeted temperature management, Therapeutic hypothermia, Traumatic brain injury, Ischemia, Reperfusion, Intracranial pressure

## Abstract

Traumatic brain injury (TBI) is recognized as the significant cause of mortality and morbidity in the world. To reduce unfavorable outcome in TBI patients, many researches have made much efforts for the innovation of TBI treatment. With the results from several basic and clinical studies, targeted temperature management (TTM) including therapeutic hypothermia (TH) have been recognized as the candidate of neuroprotective treatment. However, their evidences are not yet proven in larger randomized controlled trials (RCTs). The main aim of this review is thus to clarify specific pathophysiology which TTM will be effective in TBI.

Historically, there were several clinical trials which compare TH and normothermia. Recently, two RCTs were able to demonstrate the significant beneficial effects of TTM in one specific pathology, patients with mass evacuated lesions. These suggested that TTM might be effective especially for the ischemic-reperfusional pathophysiology of TBI, like as acute subdural hematoma which needs to be evacuated. Also, the latest preliminary report of European multicenter trial suggested the promising efficacy of reduction of intracranial pressure in TBI.

Conclusively, TTM is still in the center of neuroprotective treatments in TBI. This therapy is expected to mitigate ischemic and reperfusional pathophysiology and to reduce intracranial pressure in TBI. Further results from ongoing clinical RCTs are waited.

## Introduction

In the USA, an estimated 1.4 million people still suffer a traumatic brain injury (TBI) each year [1]. About 50,000 people die before the hospital, and at least 5.3 million live with severe disabilities related to TBI [2]. TBI thus has been a significant and growing public health issue.

The most important factor which determines the prognosis of TBI patients is the severity of the primary brain injury [3]. Additional delayed secondary brain damage is set in progress and continues from the time of traumatic impact in TBI patients, and the two combine to determine outcome [4].

Primary brain injury itself is mostly not amenable to treatment; consequently, the strategy of primary TBI treatment should be prevention, such as use of helmets and vehicle modification. Therefore, the main stream of treatment strategy for TBI should be the surgical management of TBI and neurointensive care to prevent additional secondary brain injury.

To mitigate the secondary brain injury in TBI patients, many basic and clinical researches have been performed for the innovation of pharmacological treatments and temperature managements [3, 5–7].

With the results of numerous previous basic research and clinical trials, targeted temperature management (TTM) including therapeutic hypothermia (TH) has been recognized as the candidate of neuroprotective treatment in the neurocritical care [8, 9]. However, their clear evidences in TBI patients are not yet proven in large randomized controlled trials (RCTs). TTM for TBI is thus still limited to an optional recommendation (level 3 in Brain Trauma Foundation guideline) [10].

The main aim of this review is to clarify specific pathophysiology for which TTM will be most effective. First, we will mention the general classification of pathophysiology in TBI, and we then will discuss the specific pathophysiology which will be most beneficial with TTM. In the latter part of this review, we will focus on the appropriate timing, length, and the rewarming rate of TTM in TBI patients.

## Review

### Definition of “Targeted temperature management” and “Therapeutic hypothermia”

To maintain normal physiology and to cure pathophysiology in critically ill patients, control of systematic body temperature has been enlightened in neurocritical care settings. However, several terms and definitions surrounding therapeutic body temperature management have also been existed, like TTM, TH, and therapeutic normothermia. In a review of Polderman, “hypothermia” was proposed to be defined as the status of patients’ core temperature <36.0 °C regardless of the cause. Also, “induced hypothermia” was defined as “intentional reduction of a patients’ core temperature below 36.0 °C”. Further, TH was defined as “Controlled induced hypothermia with the potentially deleterious effects such as shivering, being controlled or suppressed” [5]. On the other hand, TTM is widely including the concept of TH and therapeutic normothermia therapy. A recent report recommends that the term “Targeted temperature management” should replace “therapeutic hypothermia” [11]. In this report which was published from professional societies including the Society of Critical Care Medicine, the term “therapeutic hypothermia” was discarded in favor of TTM with emphasizing the importance of defining a complete temperature profile [11]. According to this recommendation, we also generally define and use the term “TTM” which means temperature management therapy including both of TH and therapeutic normothermia therapy in this review.

### Pathophysiology of TBI

As mentioned above, the pathophysiology of TBI is mainly divided as primary and secondary brain injuries [12]. Both primary and secondary brain injuries can be further classified by focal or diffuse mechanisms (Table 1). The distinction of focal and diffuse injuries is historically derived from the absence or presence of radiographic mass lesions on computed tomography [13]. This distinction has now evolved to consider the pathological mechanisms imparted by the trauma in regions local to and remote from the point of impact. Although these classifications are widely accepted, most TBIs consist of a heterogeneous admixture of focal and diffuse damage [12]. Focal and diffuse pathological processes are often intermingled, making it difficult to divide into focal, diffuse, and primary and secondary categories; it is useful to consider them separately for the purpose of understanding the pathophysiology (Table 1).

**Table 1:** Type and pathophysiology of traumatic brain injury

	Diffuse brain injury	Focal brain injury
Primary brain injury	• Diffuse axonal injury • Petechial white matter hemorrhage with diffuse vascular injury	• Focal cortical contusion • Intracerebral hemorrhage • Extracerebral hemorrhage (i.e., ASDH, AEDH)
Secondary brain injury	• Delayed neuronal injury • Diffuse brain swelling • Diffuse ischemic injury • Diffuse hypoxic injury • Diffuse metabolic dysfunction	• Delayed neuronal injury • Focal brain swelling • Focal ischemic injury • Focal hypoxic injury • Regional metabolic dysfunction

*ASDH* acute subdural hematoma, *AEDH* acute epidural hematoma

For example, acute subdural hematoma (ASDH) is a good representative of focal brain injury which also has the aspect of both of primary and secondary brain injuries. In ASDH, neuropathologic study showed ischemic brain damage in the hemisphere underlying the hematoma [14]. An important factor leading to this ischemic damage is raised intracranial pressure (ICP) producing impaired cerebral perfusion. Increasing ICP reduces the volume of cerebral blood circulation. Removal of the hemorrhage may result in the immediate reversal of global ischemia. And this abrupt reduction of mass lesion sometimes induces secondary “reperfusion injury” [14–16]. Previous experimental and clinical studies thus have shown that subdural hematoma and its removal was considered as an ischemic/reperfusion (I/R) pathophysiology in TBI [17, 18].

### History and future direction of TTM for TBI

Historically, TTM were induced prior to surgery to assist procedures that caused prolonged ischemia, including open heart surgery [19, 20] and various organ transplants [21]. Within its first decade, hypothermia was applied to multiple emergency situations that were characterized by ischemia such as stroke [22, 23], myocardial infarction [24], and cardiac arrest [25, 26].

As we mentioned previously, basic and clinical studies relating the effectiveness of TTM on the neuroprotective effect was also reported in TBI patients [27–29]. In 2001, a larger multicenter trial of hypothermia for neuroprotection in TBI was reported [30] (Table 2). In this RCT, 392 patients with acute brain injury were randomized to normothermia or surface cooling-induced hypothermia. Contrary to the previous phase 2 trial [27], this study could not prove the efficacy of hypothermia in TBI. However, there was a weak evidence of improved outcomes in patients who were initially hypothermic on admission and treated with continued hypothermia for 24 h [30]. This same study group then tried to confirm the efficacy of very early hypothermia in patients with severe brain injury, the National Acute Brain Injury Study:Hypothermia II (NABIS:H II) [31]. In this NABIS:H II, the early-induced hypothermia did not have efficacy when mortality and morbidity data were looked at. On the other hand, in a sub-populational analysis dividing the patients into those with diffuse brain injury and those with surgical hematoma evacuation, early-induced hypothermia proved significantly efficacious for the latter group [31]. Authors concluded that one explanation was the different pathophysiology between diffuse brain injury and hematoma. These results suggested the efficacy of TTM especially in focal brain injury which received hematoma evacuation and which had the I/R pathophysiology.

**Table 2:** Recent randomized clinical trials (RCTs) relating TTM on TBI

RCTs	Age (years old)	No. of patients	Type of TBI	Control temperature	Time interval of temperature control	Rewarming speed	Neurologic outcome	Mortality	Comments/references
NABIS:H	16–65	392	All, severe	33 °C vs 37 °C	48 h	0.5 °C/2 h	57 % poor outcome in each group, NS	28 % TH vs 27 % Normo, NS	Clifton et al. [30]
									Weak evidence of improved outcomes in patients who were initially hypothermic on admission
NABIS:H II	16–45	97	All, severe, 2.5 h after suffering TBI	33 °C vs 37 °C	48 h	0.5 °C/2 h	60 % TH 57 % Normo, NS	23 % TH vs 18 % Normo NS	Clifton et al. [30]
									Early-induced hypothermia proved significantly efficacious for surgically evacuated hematoma
B-HYPO	15–70	148	All	32-34 °C vs 35.5–37 °C	>72 h and	<1 °C/day	Relative risk (RR) 1.24, 95 % confidence interval (CI) 0.62–2.48, *p* = 0.597, NS	(RR 1.82, 95 % CI 0.82–4.03, *p* = 0.180) NS	Maekawa et al. [33]
									Clinical Trial gov. NCT00134472 UMIN 000000231
EUROTHERM 3235	−65	1800	Primary closed TBI with raised ICP >20 mmHg	32-35 °C vs Normo	48 h continued for as long as is necessary to reduce and maintain ICP <20 mmHg	NM	–	–	Andrews et al. [89]
LTH-1	18–65	300	All, GCS4-8	Longer TH (34–35 °C) for 5 days vs Normo (36–37 °C).	5 days	<0.5 °C/4 h	–	–	Lei et al. [62]
									ClinicalTrials.gov Identifier: NCT01886222
HOPES	21–65	120	ASDH with Evacuated (GCSM <6)	33 °C vs 37 °C Preoperative induction	48 h	0.1 °C/h	–	–	ClinicalTrials.gov NCT02064959 and UMIN 000014863

*TBI* traumatic brain injury, *TH* therapeutic hypothermia, *NS* not significant, *Normo* normothermia, *NM* not mentioned

The efficacy of early-induced therapeutic hypothermia was also proved in animal experimental TBI model. With considering the data of NABIS:H II, we also hypothesized that preoperatively early induced hypothermia maybe beneficial to mitigate reperfusional injury occurred by craniotomy and clot removal in ASDH rat model [32]. Our data suggested that early, preoperatively induced hypothermia could mediate the reduction of neuronal and glial damage in the reperfusion phase of I/R TBI [32].

More recently, Maekawa et al. compared prolonged mild TH versus fever control with tight hemodynamic monitoring and slow rewarming in patients with severe traumatic brain injury with a multicenter RCT (B-HYPO) in patients with severe TBI [33] (Table 2). Patients were assigned to either therapeutic hypothermia (32–34 °C) or fever control (35.5–37 °C). Patients with therapeutic hypothermia were cooled as soon as possible for ≥72 h and rewarmed at a rate of <1 °C/day. There were no significant differences in the likelihood of poor neurological outcome or mortality between the two groups. However, one subanalysis of this study showed the efficacy of hypothermia especially for young TBI patients who had focal hematoma which needed evacuation [34].

Conclusively, large RCTs still have not yet shown the efficacy of TTM in TBI treatment (Table 2). However, subanalysis of RCTs and animal experimental research showed that early, preoperatively induced hypothermia may mediate the reduction of neuronal and glial damage in the reperfusion phase of focal brain injury which has I/R pathophysiology [4].

Now, an international multicenter RCT (HOPES Trial) is currently in progress. In this trial, nine Japanese centers and three centers in the USA are included as participants. The objective of this trial is to test whether hypothermia improves the outcome following TBI with ASDH requiring evacuation. The primary objective is to determine if rapid induction of hypothermia prior to emergent craniotomy for ASDH will improve the outcome as measured by Glasgow Outcome Scale-Extended (GOSE) at 6 months. Over 120 ASDH patients will be registered by 2018 (ClinicalTrials.gov NCT02064959 and UMIN 000014863).

### The mechanisms of I/R brain injury and hypothermia treatment

Despite much research, the exact mechanisms of the I/R injury itself remain unclear. Reperfusion following ischemia can cause neurovascular injury leading to detrimental changes in the blood-brain barrier (BBB) permeability, cerebral edema, brain hemorrhage, and neuronal death by apoptosis/necrosis [35]. These complications clearly limit the benefits of reperfusional therapies. The processes leading to cellular damage after I/R injury are complex and multifactorial. At this point, the pathology of I/R injury has been separated into two distinct mechanisms. One is the cell death following cellular dysfunction, i.e., excitotoxicity, acidotoxicity, and ionic imbalance. This first process is seen primarily in the ischemic phase. The other type of injury comes from free radical production, and this becomes particularly bad during the reperfusion phase [36]. Together, these mechanisms create a complicated picture of injury (Fig. 1). In the ischemic phase, brain ischemia initiates a cascade of destructive and often irreversible processes that destroy brain cells and tissue. One example of this is the intracellular conversion to anaerobic metabolism [37]. Depletion of adenosine triphosphate (ATP) in the absence of oxidative metabolism leads to failure of the Na^+^/K^+^ ATPase pump. This causes depolarization of the cell membrane leading to activation of voltage-gated calcium channels and an influx of intracellular calcium [38]. Moreover, with the anaerobic metabolism induced, intracellular and extracellular acidosis contributes to the calcium influx. This rapid increase in intracellular calcium causes release of large amounts of the excitatory neurotransmitter glutamate, which further stimulates calcium influx in postsynaptic cells [39]. In addition to the above, calcium triggers activation of phospholipase, nitric oxide synthase, proteases, endonucleases, and oxidase enzymes [40]. These activated molecules can easily damage other cell proteins and lipid membranes causing necrosis [41]. Furthermore, recent studies have demonstrated the production of superoxide radicals by *N*-methyl-D-aspartate (NMDA) receptor-mediated nicotinamide adenine dinucleotide phosphate (NADPH) oxidase activation [42]. Such events amplify reactive oxygen species (ROS) production, mitochondrial dysfunction, and proapoptotic protein activation. Intracellular calcium accumulation itself also triggers initiation of mitochondrial dysfunction and fragmentation leading to activation of proapoptotic proteins such as the caspases [43].

**Fig. 1:** The schema of mechanisms of ischemic/reperfusional (I/R) brain injury and the effective point of hypothermia treatment. The pathology of I/R injury is approximately separated as two mechanisms, i.e., the cell death following cellular dysfunction in ischemic phase and the free radical production in reperfusion phase. The *boxed arrow* with entered “Hypothermia” means the estimated effective points in I/R cascade

Reperfusion to this ischemic tissue results in a short period of excessive free radical production [44]. Experimental measurements of the reperfusion phase demonstrate that oxygen- and carbon-centered free radicals peak within 5 min of reperfusion [45] and that hydroxyl generation peaks within 15 min [46]. This oxidative stress can damage proteins, lipids, and DNA, possibly leading to necrosis and apoptosis [47, 48]. Oxidants also modulate neuroinflammation [49] leading to increased levels of neuronal apoptosis in adjacent cells [50–52].

Despite much basic and clinical research using hypothermia in I/R brain injury, the mechanisms of its neuronal protection remain unclear. Most believe it to act through a multitude of different pathways. Mitochondrial free radical production might be an important target, and it provides a possible window of opportunity for hypothermia treatment. Supporting this point, hypothermia has been shown to decrease abnormal production of free radicals [53]. Another potential mechanism of hypothermia involves reduction of the inflammatory cascade and cell death pathways of apoptosis and necrosis [54].

Hypothermia also reduces cellular metabolism and oxygen demand while maintaining acceptable ATP levels [55]. Likewise, it improves cellular ion handling and cellular pH balance [37]. In Fig. 1, we illustrate the schema of mechanisms of I/R injury and the estimated points where hypothermia treatment can effect.

### How soon is the induction of TTM in order to be beneficial for brain injury?

The previous studies have shown that hypothermia must be achieved within 2 to 6 h of severe hypoxic-ischemic injury in animal models. For example, cooling sheep to 34 °C for 72 h gave good neuroprotection if started 90 min after the injury. It was partly effective if started at 5.5 h and was ineffective if started at 8.5 h [56]. Most clinical trials have suggested that the earlier mild hypothermia is initiated, the more likely beneficial effects may be obtained [30]. Hypothermia is currently being induced by surface cooling with use of cooling blankets, which usually requires 4 to 8 h to get the target hypothermia temperature (33 to 35 °C) [30, 57–59].

Bernard et al. reported that cooling can be achieved more rapidly (2 °C over 30 min) by intravenous administration of iced (4 °C) crystalloid solution [59].

Innovation of cooling device also enables rapid induction of TTM in TBI. Recently, the use of intravascular cooling device was spreading in the scene of neurocritical care. This device is now also approved in Japan and widely started to use for TTM in neurocritical care patients. Several reports that compare intravascular cooling to surface cooling exist. de Waard et al. compared the intravascular cooling device and surface cooling device and concluded that time to reach target temperature and cooling speeds was the same between two devices. And the variation coefficient for temperature during maintenance was higher in the surface than that for the intravascular cooling group (mean 0.85 % versus 0.35 %, *p* < 0.0001) [60]. This use of cold intravenous fluids and new cooling devices may represent a logical strategy for future clinical trials for accurate TTM in severe TBI.

### Therapeutic window for TTM

There are still no clear evidences on the optimal length of TTM in TBI. A recent experimental research showed that persisting lower temperature significantly reduced the synthesis of hypoxia-inducible factor 1 (HIF-1, a protein relating hypoxic tolerance) under hypoxic conditions and weaken adaptation to hypoxia [61]. On the other hand, a clinical research showed the efficacy of longer hypothermia therapy for neuroprotection in TBI. Jiang et al. performed a single center randomized study to compare the effect of long-term (5 days) mild hypothermia versus short-term (2 days) mild hypothermia suggesting that mild hypothermia may improve the outcome in a series of 215 severe adult TBI patients, when cooling is maintained for longer than 48 h [57]. More recently, a multicenter RCT to examine the efficacy and safety of long-term mild hypothermia (34–35 °C for 5 days) in severe TBI is planned in China (the LTH-1 trial) [62].

Rate of rewarming is also an important variable for influencing the protective effects of the hypothermia therapy. In the experimental setting, posttraumatic hypothermia followed by slow rewarming appears to provide maximal protection in terms of traumatically induced axonal damage, microvascular damage and dysfunction, and contusional expansion [63, 64]. In contrast, hypothermia followed by rapid rewarming not only reverses the protective effects associated with hypothermic intervention but also, in many cases, exacerbates the traumatically induced pathology and its functional consequences [64–66].

Conclusively, longer maintenance and slower rewarming may be beneficial in TBI. On the other hand, we also need to be cautious for severe side effects of longer hypothermia maintenance [37].

### Preoperative-induced hypothermia for traumatic brain injury

As we mentioned above, recent clinical studies suggested that preoperatively early induced hypothermia maybe beneficial in focal mass TBI. However, we still cannot find feasibility of pre- and intraoperatively induced hypothermia especially for TBI. There are some reports that used intraoperative hypothermia in neurosurgical procedures involving craniotomy (Table 3) [67–73]. These studies can teach us important lessons in planning future clinical trials using early-induced hypothermia in TBI. Specifically, we have learned that (1) perioperative-induced hypothermia is feasible and safe and (2) careful consideration should be used in determining the cooling and rewarming durations. All previous hypothermia studies describe no severe complications from the perioperative-induced hypothermia. One should note that their cooling and rewarming durations were all relatively short (Table 3). Important consideration must be given, as several researchers have pointed out, to cooling rate, period of hypothermia, rewarming rate, and volumes of intravenous fluid [74–77].

**Table 3:** Clinical studies using intraoperative hypothermia for neurosurgical procedures

Authors and year	No. of cases	Operative procedure (number)	Cooling method	Complication	Mean target temp (°C)	Mean duration of hypothermia (min)	Mean rewarming rate(°C/h)	Mean rewarming temp (°C)	Effectiveness of hypothermia
Baker et al., [67] 1994	30 (Normo 17, Hypo13 )	Elective craniotomy for supratentorial tumor resection (14), aneurysm repair (14), other (2)	WB	Shivering (Normo 0 case vs Hypo 7 cases, *p* = 0.002). No severe comp.	34.3 ± 0.4	NR	0.7 ± 0.6	35.8 ± 1.0	NR
Clifton and Christensen, [68] 1992	21 Hypo	Aneurysm surgery with elective craniotomy (21)	WB	No comp.	32.0	NR	NR	NR	NR
Hindman et al, [69] 1999	114 (Normo 57, Hypo 57)	SAH clipping (52), unruptured aneurysm clipping (62)	AC	No significant difference between Normo and Hypo. No severe comp.	33.7 (33.2–34.2)	NR	NR	35.7 (34.9–36.4)	NS
Sato and Yoshimoto [70] 2000	60 (Normo 28, Hypo 32)	SAH clipping	AC and WB	NR	34.0	NR	Time, 115 min (45–250 min)	36.2	NR
Steinberg et al., [71] 2004	153 Hypo	Elective open craniotomy for unruptured cerebral aneurysm	WB(61) vs endo(92)	Postoperative infection 4.3 % endo vs 4.9 % WB, NS. No severe comp. in all	33.0	274	1.88 (WB) vs 0.69 (endo)	(35–36)	NS between WB and endo
Todd et al, [72] 2005	1000 (Normo 501, Hypo 499)	SAH clipping	AC	Postoperative bacteremia (5 % Hypo vs 3 % Normo, *P* = 0.05, no severe comp. in all.	33.0 (32.5–33.5)	324 ± 120	NR	36.4 ± 1.0	NS
Hindman et al., [73] 2010	441 (Normo 233, Hypo 208)	SAH patients undergoing temporary clipping	AC	NR	33.3–0.8	NR	Time, 120 min	36.7–0.5	NS

*Normo* normothermia, *Hypo* hypothermia, *SAH* subarachnoidal hemorrhage, *WB* water blanket cooling, *AC* air cooling, *endo* endovascular cooling, *comp* complication, *NA*, not applicable, *NR* not reported, *NS* not significant

### Induced normothermia and avoiding hyperthermia in TBI: is it effective?

Clinical studies that prove the efficacy of induced normothermia is much less than that of induced hypothermia. One study from Pittsburgh group showed the efficacy of induced normothermia (fever prophylaxis with intravascular cooling catheter) with reduction of intracranial hypertension compared to control group [78]. More recently, Suehiro et al. reported the Japanese survey of brain temperature management (TH, intensive normothermia, and no temperature management) in patients with traumatic brain injury [79]. In this survey, a total number of 1091 patients were analyzed. Favorable outcome was significantly higher with TH group (52.4 %) compared to intensive normothermia (26.9 %) and no temperature management (20.7 %). This data suggested that TTM is significantly effective for TBI management comparing to no temperature management.

Several other studies showed that hyperthermia was associated with a statistically significant increase in the increase of ICU stay, lower Glasgow coma scale score on discharge from ICU, and lower neurological function at 6 months after initial injury [80, 81].

Conclusively, appropriate thermoregulation with TTM (TH and intensive normothermia) is significantly important in TBI. Indeed, these data have led to several recommendations for and strict control of temperature in the neuro-ICU settings [82, 83].

### TTM for controlling intracranial hypertension in TBI

Raised ICP and intracranial hypertension are important predictors of mortality in patients with severe TBI [84]. Aggressive treatment of elevated ICP has been shown to reduce mortality and improve outcome [10, 85, 86]. TTM also has been a promising treatment strategy for controlling intracranial pressure in TBI [87, 88].

To clarify the effect of TTM for the treatment of intracranial hypertension, the latest clinical trial (EUROTHERM 3235) is now ongoing [89] (Table 2). In this trial, patient with refractory intracranial hypertension (ICP > 20 mmHg) is assigned as TH group or control group (standard treatment without any TTM). Two treatment groups are compared with mortality on the 28th day after injury or on discharge. The sample size of this study is estimated as 600 patients. Recently, preliminary data of this trial showed the efficacy of TTM with controlling intracranial hypertension [90]. TTM may have a potential as a therapeutic option to control ICP in patients with severe TBI. The final result from this large RCT is waited.

## Conclusions

In this review, first, we explained the classification of TBI pathophysiology. Then, we mentioned the possibility of mild therapeutic hypothermia with focusing on the treatment of I/R-related TBI and intracranial hypertension. With considering previous RCTs, now several multicenter clinical trials including HOPES, EUROTHERM3235, and LTH-1 trial are ongoing. Conclusively, TTM is still in the center of neuroprotective treatments in TBI. These therapies are expected to mitigate ischemic and reperfusional pathophysiology and to reduce intracranial pressure in TBI. Further results from these ongoing clinical RCTs are waited.
